The article "Astragali Radix Isoflavones Synergistically Alleviate Cerebral Ischemia and Reperfusion Injury Via Activating Estrogen Receptor-PI3K-Akt Signaling Pathway" was retracted in 2023. Reasons: duplicated images; concerns about the images.

# *Astragali Radix* Isoflavones Synergistically Alleviate Cerebral Ischemia and Reperfusion Injury *Via* Activating Estrogen Receptor-PI3K-Akt Signaling Pathway

**DOI:** 10.3389/fphar.2021.533028

**Published:** 2021-02-22

**Authors:** Yong Gu, Xi Chen, Shuping Fu, Wenlan Liu, Qi Wang, Ke-Jian Liu, Jiangang Shen

**Affiliations:** ^1^ Clinical Research Center, Hainan Provincial Hospital of Chinese Medicine, Haikou, China; ^2^ Department of Core Facility, The People's Hospital of Bao‐an Shenzhen, Shenzhen, China; ^3^ School of Chinese Medicine, University of Hong Kong, Hong Kong, China; ^4^ Department of Pharmaceutical Sciences, College of Pharmacy, University of New Mexico, Albuquerque, NM, United States; ^5^ Institute of Clinical Pharmacology, Guangzhou University of Chinese Medicine, Guangzhou, China; ^6^ The University of Hong Kong-Shenzhen, Institute of Research and Innovation (HKU-SIRI), Shenzhen, China

**Keywords:** astragali radix, estrogen receptor, synergism, isoflavones, neuroprotection

## Abstract

Isoflavones are major neuroprotective components of a medicinal herb *Astragali Radix,* against cerebral ischemia-reperfusion injury but the mechanisms of neuroprotection remain unclear. Calycosin and formononetin are two major AR isoflavones while daidzein is the metabolite of formononetin after absorption. Herein, we aim to investigate the synergistic neuroprotective effects of those isoflavones of *Astragali Radix* against cerebral ischemia-reperfusion injury. Calycosin, formononetin and daidzein were organized with different combinations whose effects observed in both *in vitro* and *in vivo* experimental models. In the *in vitro* study, primary cultured neurons were subjected to oxygen-glucose deprivation plus reoxygenation (OGD/RO) or l-glutamate treatment. In the *in vivo* study, rats were subjected to middle cerebral artery occlusion to induce cerebral ischemia and reperfusion. All three isoflavones pre-treatment alone decreased brain infarct volume and improved neurological deficits in rats, and dose-dependently attenuated neural death induced by l-glutamate treatment and OGD/RO in cultured neurons. Interestingly, the combined formulas of those isoflavones revealed synergistically activated estrogen receptor (estrogen receptors)-PI3K-Akt signaling pathway. Using ER antagonist and phosphatidylinositol 3-kinase (PI3K) inhibitor blocked the neuroprotective effects of those isoflavones. In conclusion, isoflavones could synergistically alleviate cerebral ischemia-reperfusion injury *via* activating ER-PI3K-Akt pathway.

## 1 Introduction

Traditional Chinese Medicine (TCM) formulas have been used to treat stroke for centuries. With complicate active compounds after absorption and metabolism of TCM formulas, it is extremely difficult to understand exact active ingredients contributing to the pharmacological effects. Therapeutic outcome is generally attributed to the synergistic effects of multiple ingredients of TCM formula but the synergisms of the ingredients are not clearly clarified. *Astragali Radix* (AR, named *Huangqi* in Chinese, the root of plant *genus Astragalus*) is one of the most frequently used herbs for stroke treatment. According to TCM theory, AR is a principle “tonic” herb with the function of invigorating *Qi* and improving blood circulation. The crude extracts of AR have antioxidant and neuroprotective effects (He et al., 2000; Liu et al., 2019). AR contains many active compounds, including saponins, polysaccharides and isoflavones, and many ingredients have neuroprotective effects (Sinclair, 1998; Yang et al., 2013). For example, Astragaloside IV revealed to protect against cerebral ischemia-reperfusion injury (Luo et al., 2004; Qu et al., 2009; Li et al., 2012; Li et al., 2013; Wang et al., 2017). AR isoflavones protected the blood-brain barrier (BBB) integrity and reduced infarction volume in experimental ischemic stroke model (Guo et al., 2012; Fu et al., 2014; Wang et al., 2018). Therapeutically, these active compounds might have synergic neuroprotective effects against ischemic brain injury but seldom study explores the synergic effects of different compounds against ischemic brain injury.

The article "Astragali Radix Isoflavones Synergistically Alleviate Cerebral Ischemia and Reperfusion Injury Via Activating Estrogen Receptor-PI3K-Akt Signaling Pathway" was retracted in 2023. Reasons: duplicated images; concerns about the images.

Isoflavones are commonly used as health food supplements for their antioxidant properties (Messina, 2010; Romani et al., 2010; Zhang et al., 2019). There are four isoflavones in *AR:* calycosin (C) and formononetin (F) as well as two glycoside form C-glycoside and F-glycoside (Ononin). Glycoside forms of isoflavones are biologically inactive but they can be transformed to non-glycoside forms after absorption (Figure 1). Through demethylation via intestine microbe, F can be transformed into daidzein (D) (Nilsson et al., 1967; Krizova et al., 2019). C, F and D represent the total functional AR isoflavones after absorption. All those isoflavones can bind to estrogen receptors (ER) and exert their estrogenic effects as “phytoestrogens” although their binding affinities and transactivation capabilities are relatively lower than 17β-estradial (Cederroth and Nef, 2009; Tang et al., 2010). Our previous study revealed that calyscosin-7-O-β-D-glucoside, a glucoside form of C in AR, afford neuroprotective effects against ischemic brain injury through non-canonical pathway of ER signaling and harboring anti-oxidative capability (Fu et al., 2014). F was reported to protect neurons against cerebral ischemia-reperfusion injury (Liang et al., 2014). It is of great interest to determine whether these active isoflavones would act synergistically to afford greater effect against cerebral ischemia-reperfusion injury.

The article "Astragali Radix Isoflavones Synergistically Alleviate Cerebral Ischemia and Reperfusion Injury Via Activating Estrogen Receptor-PI3K-Akt Signaling Pathway" was retracted in 2023. Reasons: duplicated images; concerns about the images.

**FIGURE 1:** Structures and metabolism of *AR* isoflavones. Glycoside forms of isoflavones (calycosin-7-O-β-glucoside and ononin) are biologically inactive and can be transformed to non-glycoside forms (calycosin (C) and formononetin (F)) after absorption. Formononetin is then demethylated by intestine microbe to produce daidzein (D).

In the present study, we hypothesized that AR isoflavones could play synergistic roles in protecting against cerebral ischemia-reperfusion injury through activating ER-phosphoinositide 3-kinase (PI3K)-Akt pathway. By using *in vitro* primary cultured neurons treated with oxygen-glucose deprivation (OGD) and *in vivo* cerebral ischemia-reperfusion rat models, we investigated the neuroprotective effects of C, F and D against cerebral ischemia-reperfusion injury individually and synergistically. We found that the combination of C, F and D yielded much greater neuroprotective effects than the sum of each individual isoflavones, indicating the synergistic neuroprotective effects of different isoflavones contributing to the neuropharmacological effects of AR*.*

## 2 Materials and Methods

### 2.1 Drugs and Reagents

Isoflavones including C, F and D were purchased from Forever Biotech Inc., Shanghai, China. The purity of AR isoflavones was determined with high performance liquid chromatography (HPLC) to be at >98% for C and F, and >99% for D.

### 2.2 Primary Cell Culture

Primary cultured cortical neurons were isolated from embryonic Sprague-Dawley rats (E17). After digested by 0.25% trypsin (Invitrogen, Carlsbad, CA), cells were collected and suspended in Dulbecco’s modified eagle medium (DMEM) containing 10% horse serum, 1% l-glutamine and antibiotic mixture. The resulting single cell suspensions were seeded on 24- or 6-well plates pre-treated with poly-d-lysine (Sigma, St. Louis, MO, United States). After seeded for 4 h, the culture medium was replaced with neurobasal medium containing 2% B27 supplement, 1% l-glutamine and antibiotics mixture and cell culture was maintained at 37°C and 5% CO_2_. Immunostaining of Tuj-1 (1:200, Santa Cruz, Billerica, CA), an antibody of neuron-specific beta III tubulin, was employed to identify the mature and purity which were confirmed to be over 95%. After those cells were cultured for 10 days (DIV10), many neurites from different neurons were merged, indicating the maturation of neurons. Those cells were used for following experiments.

### 2.3 *In Vitro* Experiments and Drug Treatment

We conducted both oxygen-glucose deprivation plus reoxygenation (OGD/RO) and l-glutamate induced toxicity experiments. In the OGD/RO experiments, primary cultured neurons were exposed to neurobasal medium without glucose and incubated in a hypoxia chamber (Billups-Rothenberg, Del Mar, CA, United States) perfused with a mixed gas containing 95% N_2_ and 5% CO_2_ until medium oxygen concentration reached 0.1%, which was monitored with a PA-10A paramagnetic O_2_ analyzer (Sable Systems International, Las Vegas, NV). After cells were exposed to OGD at 37°C for 4 h, the medium was replaced with normal glucose containing medium and the plates were put into normal culture condition for 20 h for reoxygenation. In l-glutamate treatment essays, primary cultured neurons were incubated with l-glutamate (8 mM, Sigma) for 6 h, in which glutathione was depleted to induce neuronal toxicity. Different dosages (1, 5, 25 μM) of C, F and D were added to cultured medium at 15 min prior to OGD/RO or l-glutamate exposure.

The article "Astragali Radix Isoflavones Synergistically Alleviate Cerebral Ischemia and Reperfusion Injury Via Activating Estrogen Receptor-PI3K-Akt Signaling Pathway" was retracted in 2023. Reasons: duplicated images; concerns about the images.

### 2.4 Lactate Dehydrogenase Release Assay

Cytotoxicity Detection Kit (Invitrogen) was used for LDH release assay. In brief, culture medium was collected and incubated with the reaction mixture for 30 min at room temperature (24°C). Cell-free medium collected from the well was used as negative control counting as zero percent. Triton-X 100-treated cell medium was used as 100% cell death control. The optical density of the solution was measured at 490 nm on a microplate reader (Model 3,350, Bio-Rad, Hercules, CA). The rates of cell death were calculated by using the formula: Cell death rate (%) = (Experimental absorbance value − culture medium absorbance value)/(Triton-X 100-treated absorbance value–culture medium absorbance value) × 100%.

### 2.5 Middle Cerebral Artery Occlusion Model and Drug Treatments

Male adult Sprague-Daweley rats (250–270 g) were obtained from Laboratorial Animal Unit, the University of Hong Kong (HKU) and University of New Mexico (UNM). All animal experiments were approved and regulated by the Committee on the Use of Live Animals in Teaching and Research, HKU and the Laboratory Animal Care and Use Committee, UNM. All efforts were made to minimize animal suffering and to reduce the number of animals used.

Rats were subjected to MCAO to induce cerebral ischemia-reperfusion as we previously described (Shen et al., 2006). Briefly, rats were anesthetized by inhalation of 5% isoflurane and maintained with 2% isoflurane in a mixture of 70% N_2_O and 30% O_2_. After vessels isolation, a 3/0 monofilament nylon suture (Johnson and Johnson, NJ) was inserted into the external carotid artery and advanced into the internal carotid artery and anterior cerebral artery to occlude the middle cerebral artery. After occlusion for 1.5 h, the suture was removed to induce reperfusion and maintained for 22.5 h. After operation, rats were transferred to intensive care incubator in which the temperature was kept at 37°C until animals woke up completely.

The article "Astragali Radix Isoflavones Synergistically Alleviate Cerebral Ischemia and Reperfusion Injury Via Activating Estrogen Receptor-PI3K-Akt Signaling Pathway" was retracted in 2023. Reasons: duplicated images; concerns about the images.

Isoflavones (C, F and D) were dissolved in dimethyl sulfoxide (DMSO) and diluted with peanut oil to the indicated working solution (20 mM) and intraperitoneally (*i.p.*) injected to rats 30 min before suture insertion for MCAO. Same volume of DMSO and peanut oil were used as vehicle control. In parallel experiments, for mechanistic study, ER antagonist ICI 182,780 or PI3K inhibitor LY-294002 was intracerebroventricularly (*i.c.v.*) injected into the rat lateral ventricle 60 min before ischemia onset. Briefly, after anaesthetization, rat was placed on a stereotaxic apparatus and fixed well. A 22 gauge, 12 mm stainless-steel guide cannula was inserted in the left lateral ventricle of the brain. The needle was inserted 4.5 mm deep, 1.5 mm lateral to sagiture and 0.8 mm posterior to bregma to reach the lateral ventricle. Then, ICI 182,780 dissolved in DMSO (1 μM, 5 μL for each rat) or LY-294002 (10 mM, 10 μL for each rat) was slowly injected into lateral ventricle and the needle was kept for at least 30 s before removal. The same volume of DMSO was used as a negative control.

### 2.6 Infarct Volume and Neurology Scores

After 24 h of reperfusion, rat brains were isolated and sliced into coronal sections followed by staining with 2,3,5-triphenyltetrazolium chloride (TTC, Sigma, St. Louis, MO, United States) at 37°C for 20 min. The ischemic area was evaluated by calculating the hemispheric lesion area with ImageJ software (ImageJ-1.38x, United States), the relative infarct volume percentage (RIVP) was calculated as RIVP = IVA/TA×100%, IVA was the total infract area of five coronal sections, TA was the total area of five sections.

Neurological function was determined by 9-scale methods containing dysfunctional paw test, postural reflex test and circling test according to a previous report (Bederson et al., 1986). Each score was summed and represented as a single overall neurological score (0–8).

### 2.7 Western Blot Analysis

Denatured protein samples were resolved on SDS-PAGE and transferred to PVDF membrane (Millipore, Billerica, MA). After blocking, membrane was incubated overnight at 4 °C with antibodies including pAkt (Ser473) (1:500, CST, Danvers, MA), Akt (1: 1,000, CST), GAPDH (1:5,000, CST). After washing, the membrane was incubated with the goat anti-mouse or anti-rabbit HRP-conjugated secondary antibodies (1:2000, Santa Cruz). Chemiluminescence detection was performed using enhanced chemiluminescence (ECL) advance western blotting detection reagents (GE healthcare, United Kingdom).

The article "Astragali Radix Isoflavones Synergistically Alleviate Cerebral Ischemia and Reperfusion Injury Via Activating Estrogen Receptor-PI3K-Akt Signaling Pathway" was retracted in 2023. Reasons: duplicated images; concerns about the images.

### 2.8 Statistical Analysis

Data were expressed as Means ± Standard Deprivation (SD). For multiple groups designed experiments, comparisons were made by using one-way analysis of variance (ANOVA) and followed by Dunnett test for two group comparisons within the multiple groups. For two groups designed experiments, comparisons were determined using unpaired Student’s *t*-test. Statistical analysis was performed in the SPSS 16.0 statistical program (SPSS, Chicago, IL, United States) in which *p < 0.05* was considered to be statistically significant.

## 3 Results

### 3.1 Isoflavones Dose-Dependently Decrease Cell Death in Primary Cultured Cortical Neurons Under Both Oxygen-Glucose Deprivation Plus Reoxygenation Experiments and l-glutamate Experiments *In Vitro*

We firstly detected neuroprotective effects of C, F, and D alone in primary cultured cortical neurons exposed to OGD/RO condition or l-glutamate challenges. In OGD/RO experiment, the primary cultured cortical neurons were subjected to 4 h of OGD followed by 20 h of reoxygenation. In l-glutamate treatment essays, the neurons were incubated with l-glutamate (8 mM) for 6 h. C, F and D at the dosages of 1, 5, 25 μM were added to cultured medium at 15 min prior to OGD/RO or l-glutamate exposures. As showed in Figure 2, both OGD/RO exposure and l-glutamate treatment induced cell death whereas pre-treatment of those isoflavones dose-dependently reduced cell death. Those results suggest that each isoflavone has neuroprotective effects.

**FIGURE 2:** Isoflavones reduced the rate of cell death in primary cultured neurons under OGD/RO or l-glutamate-challenges. Rate of cell death was determined with LDH release assay. Isoflavones including calycosin (C), formononetin (F) and daidzein (D) were added into cultured media at the indicated concentrations prior to OGD/RO or l-glutamate (Glu) exposures. **(A)** Primary cultured mature neurons (DIV10) were exposed to 4 h OGD followed by 20 h RO. **(B)** Neurons were treated with 8 mM l-glutamate for 6 h. “Veh” means vehicle control that receives same volume of dissolvent. Data were represented as Mean ± SD, *n* = 4 (*p < 0.05, ^**^ *p* < 0.01, compared to vehicle control).

### 3.2 Isoflavones Have Synergistic Effects on Inhibiting Oxygen-Glucose Deprivation Plus Reoxygenation and l-Glutamate-Induced Cell Death *In Vitro*

A previous study reported that the contents of C and F (including glucoside conjugates) in AR was at the ratio of 1:1 whereas D was undetectable in raw materials (Xiao et al., 2004). Previous pharmacokinetic study suggests that these isoflavones can be found in serum and around 50% of F would be metabolized into D and its conjugates after AR extraction is orally administrated into rats (Singh et al., 2011). Thus, we conducted experiments to address whether these isoflavones have synergistic neuroprotective effects against OGD/RO and l-glutamate-induced neuronal cell death. We designed following groups with single isoflavones including C2.5 (2.5 μM C), F2.5 (2.5 μM F) and D2.5 (2.5 μM D), and the combined isoflavones formula including C2.5/F2.5 (C/F, 2.5 μM each), C2.5/D2.5 (C/D, 2.5 μM each), F2.5/D2.5 (F/D, 2.5 μM each) and C2.5/F2.5/D2.5 (C/F/D, 2.5 μM each). Primary cultured neurons were pre-treated with each isoflavone alone or in combination prior to OGD/RO or l-glutamate treatments. We determined the reduction rates of cell death from isoflavone treatments to vehicle control. In OGD/RO experiments, treatments of isoflavones (C, F, D) individually had only a 2% reduction of cell death whereas the combined C/D and D/F groups had around 10% and combined C/D/F group had 15%, indicating the synergistic effects of those isoflavones against OGD/RO-induced cell death (Figure 3A). The synergistic effects of isoflavones were also found in l-glutamate-challenged experiments. Exposure of l-glutamate (8 mM, 6 h) induced about 45% of cell death. Individual isoflavone treatment (C, F, D) at 2.5 μM had less than 2% reduction rate of cell death while the combined C/F, C/D and D/F treatments with 2.5 μM each had 22%, 28%, and 40%, respectively, and most remarkably, the combined C/D/F treatment had 42% (Figure 3B).

The article "Astragali Radix Isoflavones Synergistically Alleviate Cerebral Ischemia and Reperfusion Injury Via Activating Estrogen Receptor-PI3K-Akt Signaling Pathway" was retracted in 2023. Reasons: duplicated images; concerns about the images.

**FIGURE 3:** Combined isoflavone treatments had synergetic neuroprotective effects against OGD/RO and l-glutamate-induced cell death. Rate of cell death was determined with LDH release assay. Individual or combined isoflavones including calycosin (C), formononetin (F) and daidzein (D) were added into cultured media prior to OGD/RO or l-glutamate exposures. **(A)** Mature neurons treated with single isoflavone (2.5 μM) or the combined isoflavones (C2.5 μM/F2.5 μM, C2.5 μM/D2.5 μM, F2.5 μM/D2.5 μM, C2.5 μM/F2.5 μM/D2.5 μM). The reduction of cell death rate was calculated. **(B)** Mature neurons were treated with single isoflavone (5 μM) or the combined isoflavones (C2.5 μM/F2.5 μM, C2.5 μM/D2.5 μM, F2.5 μM/D2.5 μM, C1.7 μM/F1.7 μM/D1.7 μM). Data were represented as mean ± SD, *n* = 3, ^*^ *p* < 0.05. The cell death rate was recorded. **(C,D)** In l-glutamate experiments, primary cultured neurons were treated with different combinations of isoflavones prior to challenging by 8 mM l-glutamate for 6 h. “Veh” represents vehicle control that receives same volume of dissolvent. L-Glu represents “L-glutamate”. Data were represented as mean ± SD, *n* = 4, **p < 0.01.

The article "Astragali Radix Isoflavones Synergistically Alleviate Cerebral Ischemia and Reperfusion Injury Via Activating Estrogen Receptor-PI3K-Akt Signaling Pathway" was retracted in 2023. Reasons: duplicated images; concerns about the images.

Those isoflavones harboring similar structure might share the same neuroprotective mechanisms. Thus, we designed the experiments with total concentration of isoflavones equivalent to 5 μM in all single or combined isoflavone groups. Consistently, the experiments yielded the similar results. The combined isoflavone groups with C/F and D/F in the ratio of 1:1 had synergistic neuroprotective effects against OGD/RO or l-glutamate-induced neuronal cell death. The combination of three isoflavones with C/F/D at 1.7 μM each showed the best neuroprotective effect among the different combinations (Figures 3C,D). These results strongly indicate that *AR* isoflavones have synergistic neuroprotective effects against OGD/RO and l-glutamate-induced cell death.

### 3.3 Isoflavones Have Synergistic Effects on Inducing ER-PI3K-Akt Pathway *In Vitro*

We next used ER antagonist ICI 182,780 to verify the synergistic effects of isoflavones on protecting neurons and activating non-classical ER signaling in both OGD/RO and l-glutamate challenging models. As shown in Figures 4A,B, the neuroprotective effects of the isoflavones alone (25 μM) and the combined isoflavones (5 μM for each isoflavone) were decreased by pre-treatment of ICI 182,780 (Figures 4C,D).

**FIGURE 4:** Combined isoflavones groups synergistically induced Akt phosphorylation and inhibited cell death against OGD/RO and l-glutamate-induced cell death via ER-PI3K-Akt pathway. **(A,B)** Primary cultured nature neurons (DIV10) were incubated with 1 μM of ER antagonist ICI182780 for 15 min before exposed to OGD/RO (4 h OGD plus 20 h RO) or l-glutamate (8 mM l-glutamate for 6 h) challenge and treated with 25 μM isoflavones treatment. Rate of cell death was determined by LDH release assay. **(C,D)** ER antagonist was added to the groups of combined isoflavones (total concentration 5 μM). **(E)** Western blot results in the expression of *p*-Akt and Akt. **(F)** Cells were pre-treated with 10 μM LY-294002 15 min before isoflavones treatment in l-glutamate challenging model. Cell lysate was collected for the Western analysis to detect the pAkt, whereas cell medium was used to determine the rate of cell death with LDH release assay. “Veh” represents vehicle control that receives same volume of dissolvent. Data were represented as mean ± SD, *n* = 3, ^*^ *p* < 0.05, n. s.: not significant.

Induction of non-genomic ER signaling pathway could activate downstream PI3K/Akt cell survival signaling (Roman-Blas et al., 2009). The ER-mediated PI3K/Akt signaling pathway plays neuroprotective roles in cerebral ischemia induced neuronal insults (Elzer et al., 2010; Gingerich et al., 2010). Activated PI3K can induce phosphorylation of Akt at Ser473. Thus, we detected pAkt Ser473 level in each single or combined isoflavones treated group. As shown in Figure 4E, the phosphorylation of Akt at Ser473 in the groups of combined isoflavones was significant higher than that of single isoflavone treatments under both l-glutamate and OGD/RO challenged experiments. The combined formula with three isoflavones yielded the highest expression level of pAkt. Pretreatment of LY-294002 (a PI3K inhibitor, 10 μM) significantly down-regulated the expression of pAkt. The LDH release assay revealed that LY-294002 reserved the effects of the combined C/D, D/F and C/D/F treatments in the l-glutamate-mediated neurotoxicity (Figure 4F). These data suggest that the activation of PI3K/Akt pathway contributes to the synergistic neuroprotective effects of isoflavones.

The article "Astragali Radix Isoflavones Synergistically Alleviate Cerebral Ischemia and Reperfusion Injury Via Activating Estrogen Receptor-PI3K-Akt Signaling Pathway" was retracted in 2023. Reasons: duplicated images; concerns about the images.

### 3.4 Isoflavones Decreased Infarct Volume and Improved Neurological Outcome in Rat Middle Cerebral Artery Occlusion Ischemia-Reperfusion Model

We then examined the neuroprotective effects of these isoflavones by using *in vivo* MCAO cerebral ischemia-reperfusion model. After the rats were subjected to 1.5 h of MCAO plus 22.5 h of reperfusion, the vehicle treatment group revealed infarct volume up to 27.93% ± 7.1%. Treatments of C, F and D (60 μmol/kg, equivalent to 17.06, 16.1 and 15.3 mg/kg) reduced the infarct volumes to 10.99 ± 6.07%, 10.76 ± 4.21% and 13.84 ± 0.95%, respectively (Figures 5A,B). The neuroprotective effects of those isoflavones on the infarction volume became no statistically significance when the MCAO rats treated with lower dosages at 20 μmol/kg, equivalent to 5.69, 5.37, and 5.1 mg/kg for C, F and D respectively (*p* > 0.05). Meanwhile, we evaluated the effects of those isoflavones on functional recovery based on behavior deficit, which is a major endpoint in clinical trials. The MCAO rats treated with 60 μmol/kg C, F, and D displayed much improved neurological behavior deficit scores than the vehicle treatment group (Figure 5C).

**FIGURE 5:** Brain infarct volume and neurology scores in rats subjected to focal ischemia and reperfusion with or without treatment of isoflavones and ER antagonist. **(A)** Brain infarct volume of each rat was assessed by 2,3,5-triphenyltetrazolium chloride (TTC) staining. **(B)** The infarct volume was evaluated by calculating the hemispheric lesion area with ImageJ software and presented as bar graph. **(C)** Neurology score is the sum of scores of dysfunctional paw test, postural reflex test and circling test. Data were represented as mean ± S.D., *n* = 6 (^*^ *p* < 0.05). **(D,E)** Rats were intracerebroventricularly (*i.c.v.*) injected with ICI 182780 (1 μM, 5 μL) 1 h and intraperitoneally (*i.p.*) treated with isoflavones 30 min, respectively, before onset of ischemia. 24 h later, rat brains were stained with TTC and quantified (*p < 0.05, *n* = 5). “Veh” represents the vehicle control with the MCAO rats received same volume of dissolvent for isoflavones or ICI 182780. Veh/Veh represents the MCAO rats were subjected the same volume of dissolvents for both isoflavones and ICI 182780.

The article "Astragali Radix Isoflavones Synergistically Alleviate Cerebral Ischemia and Reperfusion Injury Via Activating Estrogen Receptor-PI3K-Akt Signaling Pathway" was retracted in 2023. Reasons: duplicated images; concerns about the images.

We then investigated whether ER antagonist ICI 182780 would block the synergic neuroprotective effects of those isoflavones. Rats were *i. c.v.* injected with ICI 182780 at 1 h before undergoing cerebral ischemia-reperfusion. TTC staining imaging (Figure 5D) and quantitative data (Figure 5E) showed that co-treatment of ICI 182780 partially blocked the neuroprotective effects of C and F on reducing infarct volume in the MCAO ischemia-reperfused rats. These *in vivo* animal experimental results are consistent with *in vitro* cellular experiments.

### 3.5 Isoflavones Synergistically Protect Against Cerebral Ischemia-Reperfusion Injury via Activating PI3K-Akt Signaling Pathway

We next investigated the synergistic effects of these isoflavones in reducing infarction volume in the *in vivo* MCAO model with the same protocol. As shown in Figures 6A,B, low dosage at 20 μmol/kg of C (C20, equivalent 17.06 mg/kg), F (F20, equivalent 16.1 mg/kg) and D (D20, equivalent 15.3 mg/kg) had no effect on infarction volume. However, the MCAO rats treated with the combined isoflavones, such as C10/F10 (10 μmol/kg C plus 10 μmol/kg F), had significantly lower infarct sizes than the rats treated C or F alone at the dosage of 20 μmol/kg (C20 or F20). Furthermore, the combined treatment of C, F and D with 6.67 μmol/kg each showed the best neuroprotective effects among the groups. These results suggest that the combined isoflavones formula could synergistically decrease infarct volume against cerebral ischemia-reperfusion injury.

**FIGURE 6:** The infarct volume of the brains from MCAO rats received single or combined isoflavones treatment with or without PI3K inhibitor treatment. **(A)** The representative images of infarct brain sections in the rats treated with different combined isoflavones of calycisin (C), formononetin (F) and daidzein (D). **(B)** Infarct size in each group was calculated with ImageJ. Data were represented as mean ± S.D., *n* = 5 in C20, D20 and C10/F10; *n* = 4 in Veh and F20; *n* = 6 in C10/D10, D10/F10 and C6.67/F6.67/D6.67 (^*^ *p* < 0.05) **(C,D)** Rats were *i.c.v.* injected with LY294002 (10 mM, 10 μL) or vehicle control 60 min before onset of ischemia in C/F/D-mediated synergistic neuroprotective model. “Veh” represents the vehicle control with the MCAO rats received same volume of dissolvent for isoflavones **(A,B)** or LY294002. Data were represented as mean ± SD, *n* = 6, ^*^ *p* < 0.05.

The article "Astragali Radix Isoflavones Synergistically Alleviate Cerebral Ischemia and Reperfusion Injury Via Activating Estrogen Receptor-PI3K-Akt Signaling Pathway" was retracted in 2023. Reasons: duplicated images; concerns about the images.

We finally used PI3K inhibitor LY-294002 to investigate whether AR isoflavones synergistically regulate PI3K-Akt signaling pathway. As C, F and D combination yielded the best neuroprotective effects, we selected the combined formula of C/F/D to understand the mechanism of synergism. LY-294002 (CFD-LY) were *i.c.v.* injected into the rats before the combined C/F/D treatment. As shown in Figures 6C,D, pretreatment of LY-294002 significantly reduced the effects of combined C/F/D treatment on infarct volume. These results indicate that AR isoflavones have the synergistic neuroprotective effects through activating PI3K/Akt signaling pathway.

## 4 Discussion

To the best of our knowledge, this is the first report demonstrating the synergistic neuroprotective effects of different isoflavones with similar parent structure against cerebral ischemia-reperfusion injury. *AR* isoflavones synergistically regulated ER-PI3K-Akt signaling pathway and subsequently protected neurons from cerebral ischemia-reperfusion injury.

*Astragali Radix* is the most representative herb used for stroke treatment. Isoflavones are its representative neuroprotective ingredients. Previous studies by us reported that calycosin and its glucoside derivatives have neuroprotective effects against cerebral ischemia-reperfusion injury (Guo et al., 2012; Fu et al., 2014). Thus, we selected C and F and their metabolite D, and investigated their synergic neuroprotective effects against cerebral ischemia-reperfusion injury. The combined formula with C/D, F/D and C/F/D had remarkably enhanced neuroprotective effects when compared with individual isoflavones at same doses in the OGD/R and l-glutamate-induced neurotoxicity *in vitro* and MCAO cerebral ischemia and reperfusion injuiry *in vivo*. The C/F/D group yielded the best outcomes, indicating the synergistic protecting neuroprotective effects of those isoflavones. Notably, although they are isoflavone derivatives with similar parent chemical structures, the combination strategy of the isoflavones revealed the neuroprotective effects superior to individual isoflavone with equivalent concentration. Those results strongly support that isoflavone derivatives have synergic neuroprotection against cerebral ischemia-reperfusion injury.

Estrogen has neuroprotective effects against neuronal cell death via binding and activating estrogen receptor. The neuroprotective effects of estrogens have been reported in the *in vitro* experimental neurotoxic models, such as glutamate excitotoxicity (Goodman et al., 1996; Singer et al., 1999; Gingerich et al., 2010) and OGD-induced neuronal cell death (Harms et al., 2001; Cimarosti et al., 2005), and the *in vivo* models of cerebral ischemia injury (Simpkins et al., 1997; Dubal et al., 1998; Lebesgue et al., 2010). The neuroprotective mechanisms could be related to non-genomic estrogen signaling other than canonical estrogen signaling pathway (Pupo et al., 2016; Ranganathan et al., 2019). For 17β-estradiol-mediated neuroprotection, the ligand binds to ERα, β and GPR30, and activates the downstream survival signaling such as MAPK (Jover-Mengual et al., 2007; Zhao and Brinton, 2007), STAT3 (Dziennis et al., 2007), and PI3K/Akt (Cimarosti et al., 2005). Herein, we found that ER antagonist and PI3K inhibitor partially reversed the neuroprotective effects of isoflavones either in individual isoflavone and combined *AR* isoflavones. Those partial abolition of the neuroprotective effects of isoflavones might be explained by the incomplete blockade on the isoflavone-induced ER activation by ICI 182,780. Other possible explanation is that the antioxidant properties would also contribute to the neuroprotection of these isoflavones. Our previous study revealed isoflavones could regulate nitric oxide/caveolin-1/matrix metalloproteinases pathway and protect blood-brain barrier integrity in experimental cerebral ischemia-reperfusion injury (Fu et al., 2014). Nevertheless, current study suggests that the isoflavones-mediated ER signaling pathway contributes to the neuroprotective effects.

The article "Astragali Radix Isoflavones Synergistically Alleviate Cerebral Ischemia and Reperfusion Injury Via Activating Estrogen Receptor-PI3K-Akt Signaling Pathway" was retracted in 2023. Reasons: duplicated images; concerns about the images.

Our data showed that the *AR* isoflavones activated the ER-PI3K-Akt pathway, which partly explains the mechanisms of the synergistic roles of the isoflavones for neuroprotection. Following points could explain the underlying mechanisms of the synergism: 1) Isoflavones bind to ER with different binding affinity, but the binding sites are unclear yet. Binding of one isoflavone could change the ER structure state and increase the binding affinity to other isoflavone, which is namely allosteric effect. 2) Phytoestrogens can alter the expression of estrogen receptors. Genistein showed to increase the expression of ERα in ovary (Jefferson et al., 2002). Daidzein enhanced the expression of ERα and ERβ at both mRNA and protein levels in granulosa cells (Nynca et al., 2009). Perinatal mice treated with daidzein displayed the elevated ERα expression in the brains (Yu et al., 2013). Therefore, C, F and D might promote ER expression and produce more binding sites for isoflavones, thereby providing the synergistic neuroprotective effects. 3) Isoflavones have anti-oxidative and/or iron-binding effects.

The article "Astragali Radix Isoflavones Synergistically Alleviate Cerebral Ischemia and Reperfusion Injury Via Activating Estrogen Receptor-PI3K-Akt Signaling Pathway" was retracted in 2023. Reasons: duplicated images; concerns about the images.

In addition, the combination of dietary or herbal phytoestrogens with diverse molecular mechanisms may also enhance their efficacy. For instance, it has been reported that the combination of any two or three of genistein, quercetin and biochanin A synergistically enhanced the chemotherapeutic effects against prostate cancer and improved the efficacy at physiologically achievable concentrations (Kumar et al., 2011). Genistein and daidzein, two soy isoflavones, revealed the synergic protective effects against UVB-induced DNA damage (Iovine et al., 2011). Therefore, the synergistic effects of isoflavones could exist in different pathological and physiological conditions. The other possible explanation would be that the combined isoflavones could synergistically activate other signaling pathways for neuroprotection in ischemic/hypoxic neurons whereas individual isoflavones would have no such synergism.

The combination of three isoflavones displayed different extent of infarct size reduction in two experimental designs (Figures 6A–D). This inconsistency of infarct sizes often happened in experimental stroke rat models when different batches of animals subjected to the similar surgical protocols. There are two plausible explanations to the inconsistency. First, these two parts of experiments were conducted in different time using different batches of rats. The different populations of animals might have different responses to the vehicle treatment and ischemia. Second, intracerebroventricularly injection of 1 μM DMSO (used as the vehicle control for LY-294002) in the rats of latter design might bring additional injury to increase the infarct size.

There is a critical limitation of our present research. The doses of isoflavones used in the study of synergistic neuroprotection are comparatively low and single. This may affect the fact that whether these isoflavones can also have synergistic neuroprotective effects in other dose ranges. More doses and combinations of these isoflavones should be employed in future studies to confirm their synergism.

In conclusion, AR isoflavones synergistically protect neurons against ischemia-reperfusion injury *in vivo* and *in vitro* and the ER-PI3K-Akt pathway is likely the molecular target of AR isoflavones contributing to their synergistic neuroprotection. The discovery of the synergistic effects of the combination strategy of isoflavone derivatives brings better understanding the neuroprotective mechanisms of isoflavones against cerebral ischemia-reperfusion injury. Importantly, the study opens a new window for developing the therapeutic strategy for better outcome in the treatment of ischemic stroke.

The article "Astragali Radix Isoflavones Synergistically Alleviate Cerebral Ischemia and Reperfusion Injury Via Activating Estrogen Receptor-PI3K-Akt Signaling Pathway" was retracted in 2023. Reasons: duplicated images; concerns about the images.

## Data Availability

All datasets generated for this study are included in the article/supplementary files.
